# Deep Learning-Based Image Automatic Assessment and Nursing of Upper Limb Motor Function in Stroke Patients

**DOI:** 10.1155/2021/9059411

**Published:** 2021-08-24

**Authors:** Xue Chen, Yuanyuan Shi, Yanjun Wang, Yuanjuan Cheng

**Affiliations:** ^1^Department of Orthopedics, The Second Hospital of Jilin University, Changchun 130041, China; ^2^Department of Nursing, The Second Hospital of Jilin University, Changchun 130041, China

## Abstract

This paper mainly introduces the relevant contents of automatic assessment of upper limb mobility after stroke, including the relevant knowledge of clinical assessment of upper limb mobility, Kinect sensor to realize spatial location tracking of upper limb bone points, and GCRNN model construction process. Through the detailed analysis of all FMA evaluation items, a unique experimental data acquisition environment and evaluation tasks were set up, and the results of FMA prediction using bone point data of each evaluation task were obtained. Through different number and combination of tasks, the best coefficient of determination was achieved when task 1, task 2, and task 5 were simultaneously used as input for FMA prediction. At the same time, in order to verify the superior performance of the proposed method, a comparative experiment was set with LSTM, CNN, and other deep learning algorithms widely used. *Conclusion*. GCRNN was able to extract the motion features of the upper limb during the process of movement from the two dimensions of space and time and finally reached the best prediction performance with a coefficient of determination of 0.89.

## 1. Introduction

Cerebral apoplexy (CA), also known as cerebral stroke or cerebral vascular accident (CVA), is a kind of acute cerebrovascular disease and is due to the sudden rupture of blood vessels in the brain or due to blood circulation obstruction caused by blood vessel damage caused by a group of diseases. Stroke is one of the three major diseases leading to human death. It has the characteristics of high morbidity, high mortality, high disability, and high recurrence rate. China is a region with a high incidence of stroke. According to the data of “2018 China Health Statistics Summary,” in 2017, the proportion of cerebrovascular diseases in the deaths of Chinese residents was 23.18% in the rural population and 20.52% in the urban population, which means that at least one person in every five deaths died from stroke. According to the 2018 Report on Stroke Prevention and Treatment in China, the number of stroke patients in residents over 40 years old has reached 12.42 million, and since 2002, the incidence of the first stroke in residents between 40 and 74 years old has increased by 8.3% on average every year, and the number of deaths caused by stroke has reached 1.96 million every year. Stroke has overtaken diseases such as ischemic heart disease, traffic accidents, chronic pulmonary obstruction, and lung cancer to become the leading cause of death. With the development of modern medicine, the level of treatment in the acute stage of the disease has been improved, and the number of death cases caused by stroke has gradually decreased, but the residual dysfunction has also led to a gradual increase in the rate of disability, which greatly affects the healthy life of patients and their families.

Stroke can be divided into hemorrhagic and ischemic diseases pathologically. Different clinical manifestations may occur due to different sites and properties of the lesions. 55%∼75% of surviving stroke patients will remain with limb dysfunction, and 85% of patients will have lateral limb motor dysfunction after onset. In patients with hemiplegia, the incidence of motor function injury of the half limb, especially the hand function and upper limb motor dysfunction, is higher than that of the lower limb, and its rehabilitation difficulty is higher than that of the lower limb. These functional disorders seriously affect the ability of patients to live independently and reduce the quality of life of patients. Clinical observation shows that rehabilitation treatment is the most effective way to reduce the disability rate of stroke patients. Effective rehabilitation training plays an important role in improving the motor ability, sensory ability, and behavioral ability of stroke patients. Rehabilitation training can improve the daily living ability of patients, improve the ability to recover from brain lesions, reduce the degree of disability, restore the ability of independent living, better return to family and society, reduce potential nursing costs, and save social resources.

Stroke rehabilitation is a circular process, mainly including the following links: (1) rehabilitation assessment, identification, and determination of patients' needs; (2) rehabilitation goal setting, to develop practical and achievable rehabilitation goals and health training plans for patients; (3) rehabilitation treatment to achieve rehabilitation goals; and (4) evaluation of rehabilitation again to evaluate the therapeutic effect of the rehabilitation process.

In this paper, sensor technology and artificial intelligence were integrated to carry out the research on automatic assessment of stroke upper limb motor function based on deep learning. A motion measurement system was designed from the upper limb motor ability, and three different deep learning methods were proposed to extract features based on sensor data to achieve clinical scale stages and score prediction.

Upper limb hemiplegia is one of the most serious disabling consequences of stroke [1]. There are many studies on the influence of upper limb motor function of patients. Mullick et al. discussed the influence of motion observation training based on the mirror neuron system on upper limb motor function of stroke patients [2]. Gunduz et al. aimed to investigate the influence of hand robot assisted training based on motion imagery on upper limb function of stroke patients [3]. Brewer et al. investigated the effect of high frequency repetitive transcranial magnetic stimulation (HF-rTMS) on upper limb motor function in the early stage of stroke [4]. Strippoli et al. discussed the effect of restrictive exercise therapy (CIMT) on the rehabilitation of upper limb motor function in stroke patients [5]. Simpkins et al. investigated the effect of upper limb isokinetic muscle strength training on motor function of stroke patients [6]. Liou et al. discussed the influence of mirror therapy on upper limb function and daily living ability of stroke patients with hemiplegia [7].

In order to objectively quantify the upper limb motor injuries of stroke patients with hemiplegia, Fu et al. proposed an assessment method based on motion coordination quantization and multimodal fusion. Principal component analysis (PCA) and K-weighted angular similarity (K-WAS) algorithm were used to quantify the synergistic effect and muscle synergistic effect so as to further analyze the synergistic activation characteristics leading to visible sports injuries [8].

Quantitative assessment of motor function is important for post-stroke patients because it can be used to personalize treatment strategies. Pan et al. studied the assessment method of upper limb motor function in stroke patients. During voluntary upward extension, inertial sensor data and surface electromyography (sEMG) signals were collected from the upper limb. Five features include the maximum shoulder joint angle, peak and average velocity, trunk balance calculated from inertial sensor data, and muscle cooperative similarity extracted from surface EMG data by the nonnegative matrix factorization algorithm [9]. Sang-Mi et al. used BCT to quantitatively detect the motor imaging ability of stroke patients and clarified the relationship between the motor imaging ability of the upper limb of hemiplegia, motor function, and the use level of paralyzed limbs [10].

Fusion in sensor technology and artificial intelligence in this paper, based on in-depth study of the upper limb movement function stroke automatic evaluation of research, probes into the upper limb after stroke activity ability to automatically assess the related content, including the clinical ability of upper limb activity in clinical evaluation of relevant knowledge, called sensors for upper limb bones point spatial location tracking, and GCRNN model building process.

## 2. Materials and Methods

In order to evaluate the performance of the proposed deep learning method for predicting the FMA score of upper limb motor function, Kinect V2 was selected in this paper to measure the upper limb motor function of stroke patients. Group-constrained convolutional recurrent neural network (GCRNN) is used to achieve this task. We first designed a unique experimental environment and called volunteers to complete the required data collection of upper limb skeletal map. By analyzing the correlation between the predicted value of the model and the actual evaluation score of clinicians, we verified the performance of the model in each evaluation task and the overall performance.

In order to avoid the interference of background and other external factors, improve the quality of data, and ensure the consistency, we first set up a unique experimental environment for the collection experiment of bone point position sequence required by model training. The Kinect V2 is mounted 1.5 meters away from a chair with a small armrest. The subject will sit in this chair and complete the rating task. The Kinect V2 connects to a PC via a USB cable to transfer data and instructions. When subjects performed the upper limb assessment task, Kinect collected the three-dimensional spatial location information of the upper limb bone points in the process at a frequency of 30 Hz and transmitted and stored it to the PC in real time. Before the FMA test, we adjusted the Kinect V2's installation angle so that it could track the entire upper limb of the subject.

A total of 15 healthy volunteers were recruited in this experiment, including 9 males and 6 females, with an average age of 22.6 (±1.4) years old. Each volunteer was a stroke patient whose FMA score of upper limb motor function was randomly simulated between 30 and 100 points and who could keep sitting position. The basic information of the subjects is shown in Table 1.

Subjects sit on chairs in the experimental environment by themselves and coordinate with the experimenter to adjust the posture angle for better data collection. Then, subjects need to repeat the following upper limb assessment movements successively under the guidance:

### 2.1. Shoulder Buckling

Subject will sit in a chair and raise the upper limb of the hemiplegia side as far forward as possible, hold for 5 seconds, and finally return to the starting position.

### 2.2. Shoulder Abduction

Subjects sit in a chair and extend their upper limb on the hemiplegic side as far as possible, then hold it for 5 seconds, and finally return to the starting position.

### 2.3. The Forearm before and after the Rotation

Subject is sitting in a chair with shoulder 0° and elbow 90° flexed and forearm pronated forward and backward.

### 2.4. Finger Pinch

When the shoulder of the affected side is 0° and the elbow is 90° flexed, try to touch the little finger with the thumb and then move back to the initial position.

### 2.5. Move the Cylinder Object

Use the affected hand to pick up a cylinder on one side of the table and then move it to the other side of the table and lower it.

Each rating action was provided with an instructive video, and the subjects were asked to try their best to complete the rating action (simulation) while watching the video. At the same time, two raters were responsible for rating according to the FMA requirements and experience according to the completion of the action. Then, the average of the FMA scores obtained by the two raters was calculated. The actual FMA score of the subject was used for model training. Before the experiment, each subject will watch the instruction video of learning movements and practice the familiar movements for 3–5 times before starting the experiment. During the experiment, the subjects need to complete all the 5 movements continuously with a short rest interval of 2-3 seconds to facilitate the later data separation. The subjects can repeat 3–5 times according to their own physical conditions. Cameras were also used to record the whole experiment process, measure the time required for each experiment process, and analyze the movements of the subjects.

## 3. Results and Discussion

We verify the performance of the method proposed in this paper, namely, the comparison algorithm, by using five-fold cross validation of the data set. Each method iterates 100 times in the near row of the training set, and the iteration parameter with the best performance on the validation set is taken as the final result. The model outputs were predictive FMA scores of upper limb motor function. Performance was evaluated by correlation analysis with clinician scores, and coefficient of determination (*R*^2^), root mean square error (RMSE), and adjustment-*R*^2^ were used as model performance indicators.

First, we analyzed the correlation analysis results of the proposed algorithm for the 5 scoring tasks separately, as well as the correlation analysis results of FMA prediction using the data of the 5 tasks, as shown in Figure 1, and it can be found that task 1, task 2, and task 5 have a high correlation with FMA, and the determination coefficients of 0.88, 0.85, and 0.87 can be reached when using these rating tasks alone. Because task 3 and task 4 only have local hand movements, the correlation with the overall FMA rating item is weaker. Therefore, the consistency with the clinician's FMA assessment was only 0.78 and 0.72. When we input all the bone point data of the five assessment tasks into the model for FMA prediction, as shown in Figure 1(f), although the determination coefficient obtained is improved compared with that when using single task data as input, the improvement effect is not obvious. The coefficient of determination is 0.86, which is lower than that of Task 1 (Figure 1(b)) and Task 5 (Figure 1(e)).

In order to achieve automatic upper body activity assessment using as few assessment tasks as possible, we conducted prediction performance under different number and combination of tasks in order to find the most appropriate number and combination of assessment tasks. According to the experimental results shown in Figure 1, we conducted a comparative verification experiment in accordance with some combinations that might be better. The results are shown in Table 2.

As can be seen from the table, when the task combination is Task 1-2-3-5, the maximum coefficient of determination can be reached to 0.89; when the number of tasks is 2, the overall coefficient of determination is relatively low because there are too few FMA assessment items covered and the upper limb movement features can be provided. When the number of assessed tasks was 3, compared with the number of assessed tasks was 2, there was a significant improvement, but different combination of tasks also had an impact on the experimental results. Because task 4 and task 5 were both hand functional assessments, the combination of task 4 and task 5 provided overlapping motor function characteristics. In addition, it can be seen from Table 2 that the task combination of Task 1, 2, and 5 can provide more motor characteristics from multiple dimensions such as shoulder abduction, forward bending, and grasping ability, covering more FMA assessment items.

In order to verify the performance of the proposed deep learning framework, we used the optimal combined task data of Task 1, 2, 3, and 5 mentioned above to conduct comparative experiments with the GCRNN algorithm in this paper, LSTM and CNN algorithm. Regression analysis was performed on clinician evaluation scores and model-predicted FMA scores of 15 subjects, and determination coefficients were calculated, and correlation analysis graphs were drawn, as shown in Figures 2–4. The GRCNN model fully extracts the spatial location sequence data features of bone points from the two dimensions of data sequences between data sequences and the context of a single data sequence through convolution and cyclic neural network modules and finally predicts the optimal performance when the coefficient of determination of FMA fraction reaches 0.89 (Figure 2). In the manifestation of upper limb motor dysfunction, the relationship between bone nodes in the human body can reflect the cooperative movement mode often manifested in clinical practice and so on. Compared with LSTM, CNN pays more attention to the feature extraction of the relationship between data, and in the upper limb motor ability assessment task in this paper, it also obtains a coefficient of determination of 0.87 (Figure 3). The LSTM model pays more attention to the before and after dependence of the sequence. Stroke-related patients have a small range of upper limb motion, weak features of the before and after changes in the sequence data, and relatively weak performance in automatic assessment tasks. The coefficient of determination in the data set in this paper is 0.85 (Figure 4).

IMU, glove sensor, and motion capture system often used in existing studies need quite a long time to complete the wearing and marking, and it is already difficult to fix the sensor or marker on the body of stroke patients, and it is easy to cause discomfort to patients and affect normal activities. The automatic evaluation system proposed in this paper uses the Kinect V2 depth sensor based on vision to collect motion data. It does not require the time-consuming process of sensor wearing. It only takes about 5 minutes to set up the initial (perspective setting) and has a generally acceptable low cost. The rich SDK provided by Kinect can obtain various motion tracking data, such as RGB image, depth image, and spatial position of bone points. In this paper, the spatial position data of human upper limb bone points were only used to complete the task of upper limb mobility assessment. In the future work, we can also consider the use of depth image, RGB, and combined data for automatic evaluation research. In addition, we also found that there are some insurmountable errors in acquiring it through noncontact motor consciousness in our experiment. When subjects wear loose clothes, there is a deviation in the recognition and tracking of shoulders and elbows. When human beings are active, it will bring great interference to the data. Such data patterns can be confused with data disturbances caused by limb spasms. Second, the Kinect V2 only has two bone points on the hand, the thumb, and the fingertip, which poses a huge challenge to complete the measurement of hand extension/flexion motion in FMA. In addition, when a single Kinect performs task 5: upper limb activity tracking of moving pencil and limb occlusion is easy to occur, which will cause the data loss of occluded bone points, thus affecting the accuracy. Of course, this problem of being easily obscured can be solved in the future by setting up multiple Kinect devices to track human activities from different angles.

## 4. Conclusions

The focus of this paper is to propose a deep learning framework for data analysis, to achieve the use of as few assessment tasks as possible to complete the complex clinical FMA assessment tasks, and to achieve a high degree of consistency with the clinician assessment. Through a detailed analysis of all FMA evaluation items, we set up a unique experimental data collection environment and evaluation tasks. The results of FMA prediction using bone point data of each evaluation task are shown in Figure 1. Through different number and combination of tasks, it can be seen in Table 2. The best coefficient of determination was achieved when task 1, task 2, and task 5 were simultaneously used as inputs for the FMA prediction. At the same time, in order to verify the superior performance of the proposed method, a comparative experiment was set with LSTM, CNN, and other deep learning algorithms widely used. GCRNN was able to extract the motion features of the upper limb during the process of movement from the two dimensions of space and time and finally reached the best prediction performance with a coefficient of determination of 0.89.

## Figures and Tables

**Figure 1:** Individual assessment task data predicts FMA results.

**Figure 2:** GCRNN performed FMA prediction performance.

**Figure 3:** FMA prediction performance by CNN.

**Figure 4:** LSTM performed FMA to predict performance.

**Table 1:** Subject information table.

Attribute	Value
Male	9
Female	6
Age range	21–24
FMA score range	30–100

**Table 2:** Comparison of evaluation task combinations.

Number of tasks	Task combination	RMSE	*R* ^2^	Adjust-*R*^2^
2	Task 1-2	7.29	0.86	1.19
	Task 2-5	7.30	0.86	1.21

3	Task 1-2-5	7.25	0.88	1.23
	Task 2-4-5	7.90	0.84	1.25
	Task 2-3-5	7.26	0.87	1.19

4	Task 2-3-4-5	7.81	0.85	1.24
	Task 1-2-3-5	6.57	0.89	1.17
	Task 1-2-4-5	7.40	0.86	1.22

5	Task 1-2-3-4-5	7.37	0.86	1.21

## Data Availability

The data used to support the findings of this study are available from the corresponding author upon request.
